The article "Surgical Treatment of Radiation-Induced Late-Onset Scalp Wound in Patients Who Underwent Brain Tumor Surgery: Lessons from a Case Series" was published in 2022. Journal: Biomed Res Int.

# Surgical Treatment of Radiation-Induced Late-Onset Scalp Wound in Patients Who Underwent Brain Tumor Surgery: Lessons from a Case Series

**DOI:** 10.1155/2022/3541254

**Published:** 2022-05-25

**Authors:** Jinhyun Kim, Kyung Chan Ahn, Hak Chang, Jae Hoon Jeong, Changsik John Pak, Byung Jun Kim

**Affiliations:** ^1^Department of Plastic and Reconstructive Surgery, Seoul National University Hospital, Seoul 03080, Republic of Korea; ^2^Hyundai Aesthetic Plastic Surgery, Seoul 06038, Republic of Korea; ^3^Department of Plastic and Reconstructive Surgery, Seoul National University Bundang Hospital, Seongnam 13620, Republic of Korea; ^4^Department of Plastic and Reconstructive Surgery, Asan Medical Center, Seoul 05505, Republic of Korea

## Abstract

**Objective:**

The management of late-onset scalp wounds following irradiation is troublesome, especially in patients with a surgical history of intracranial neoplasms. It, insidiously, starts with wound dehiscence or discharge and never heals spontaneously without appropriate surgical treatment. Nevertheless, definite treatment guidelines have not yet been established. Here, we present our clinical experience with radiation-induced scalp wounds and suggest a surgical principle for their treatment. *Patients and Methods*. The medical records of 13 patients with brain tumors, who were treated for intractable scalp wounds after irradiation between January 2000 and August 2015, were retrospectively reviewed. All the patients underwent a craniotomy for brain tumor resection. Surgical treatment for a late-onset scalp wound was decided based on the “reconstructive ladder” and according to the status of bone flap and scalp tissue. The patients' clinical characteristics and information regarding irradiation, surgery, and postoperative complications were recorded.

**Results:**

Scalp wounds developed 4.4 years, on average, after the completion of irradiation. Revision operations were performed an average of 2.3 times, and 6 patients (46%) required more than 2 operations. The bone flap was removed in 11 patients (84.6%) to achieve complete wound healing. Among them, 3 patients underwent a cranioplasty using artificial materials, but 2 patients underwent removal due to recurrent wound problems.

**Conclusions:**

Postirradiation scalp wounds are difficult to treat and have a high risk of recurrence. If osteoradionecrosis is suspected, the bone flap should be removed. It is important to debride unhealthy tissues aggressively and cover defects with robust tissue.

## 1. Introduction

Current treatment for intracranial neoplasms involves surgical excision combined with adjuvant chemotherapy and radiotherapy to eradicate remnant tumors. Advances in the treatment of brain tumors have improved patient survival, but the incidence of radiation-related long-term complications has also increased.

Damage to the vasculature and abnormal collagen deposition by cytokines are thought to be the main processes involved in the development of radiation-induced fibrosis (RIF) and sclerotic and atrophic tissue changes, which are considered to be late complications [1, 2]. Osteoradionecrosis (ORN) is another devastating late complication that can occur in bony tissue after irradiation. Once it develops, it is prone to infection, and conservative management is difficult [3].

Several considerations should be made when treating radiation-induced scalp wounds in patients with intracranial neoplasms. First, tumor recurrence should be ruled out as it may mimic the effect of radiation on tissues. Second, since the bone flap created during craniotomy has poor vascularity, ORN is likely to develop upon irradiation. Therefore, the appropriate management of bone flaps is essential for wound healing. Third, scalp reconstruction has a relatively high risk of complications [4, 5]. Moreover, fibrotic changes after irradiation make it harder for the scalp defect to be closed in a tension-free fashion. Therefore, conventional surgical algorithms for scalp reconstruction cannot be applied in these situations.

Previously, there have been studies on the reconstruction of scalp defects or the management of radiation-induced wounds [6, 7]. Nevertheless, there are no studies focusing on the surgical treatment of late-onset radiation-induced intractable scalp wounds in patients who underwent craniotomies for brain tumor resection. In this study, we present the lessons learned from our clinical experiences and suggest surgical principles to assist surgeons in planning treatment strategies.

## 2. Patients and Methods

This study was performed in accordance with the 1975 Declaration of Helsinki guidelines. All investigations were carried out after receiving approval from the institutional review board (approval number: H-1512-056-727), and informed consent was obtained. The medical records of 13 patients treated for late-onset scalp wounds after irradiation at our department between January 2000 and August 2015 were reviewed retrospectively. All patients underwent surgical treatment for intracranial neoplasms by neurosurgeons and received irradiation to eradicate possible remnant tumors. Patients were excluded if wound problems were caused by tumor recurrence or if they occurred within six months after irradiation.

Information, including patients' underlying diseases, surgical history of brain tumors, chemotherapy history, irradiation dose, and fraction, was recorded. Information regarding scalp reconstruction, such as the time until wounds developed after irradiation, clinical characteristics of the wounds, type of operation performed, microbial culture results, follow-up period, and postoperative complications, was also collected. Medical photographs, imaging results, and histological slides were evaluated (Table 1).

## 3. Results

Thirteen patients (7 men and 6 women) were enrolled. Patients were treated for intracranial neoplasms, such as glioblastomas, anaplastic astrocytomas, anaplastic oligodendrogliomas, atypical meningiomas, and brain metastasis. Biosynthetic materials were used to cover any dural defects caused by the tumorectomy. Lyodura® (Braun Melsungen AG, Melsungen, Germany) was used in 4 patients, and porcine submucosa Surgisis® (Cook Surgical, Bloomington, IN) was used in 1 patient. All patients received irradiation sessions with an average dose of 56.7 Gy delivered in 31.8 fractions. Scalp wounds developed 4.4 years after the completion of irradiation and presented as wound dehiscence, oozing, pus-like discharge from the wound, or excessive growth of granulation tissue.

Revision operations were done 2.3 times, on average, and 6 patients (46%) required more than 2 operations. The bone flap was removed in 11 patients (84.6%) to achieve complete wound healing. Among them, 3 patients underwent cranioplasty using artificial materials, but 2 patients underwent removal due to recurrent wound problems. The mean follow-up period was 6.6 years (Table 1).

### 3.1. Case 1 (Patient 5)

A 48-year-old male patient underwent a near-total removal of aplastic meningomyeloglioma 14 years ago, followed by adjuvant radiation therapy (total dose: 61.2 Gy). Soft tissue bulging developed recently near the previous surgical scar, which was confirmed to be inflamed granulation tissue on biopsy. An open wound developed shortly after the biopsy, which did not heal with repeated dressing for >3 months. Initially, debridement and coverage with a local rotational flap were performed, but wound breakage recurred. A secondary local flap also failed to achieve wound healing; therefore, an anterolateral thigh (ALT) [8] free flap transfer was performed, discarding the scalp tissue, which showed hardened and inelastic characteristics of RIF (Figure 1). Regardless, we eventually failed to salvage the ALT flap due to infection. Finally, the underlying bone flap was completely removed, and a second free flap was transferred using Latissimus dorsi (LD) muscle with a split-thickness skin graft (STSG). The wound healed well, without further complications (Figure 2).

### 3.2. Case 2 (Patient 7)

A 36-year-old woman had previously undergone total resection of anaplastic astrocytoma. A total radiation dose of 62.6 Gy was administered postoperatively. After 3.5 years, a pus-like discharge was noticed through a wound break, and methicillin-resistant *Staphylococcus aureus* (MRSA) was identified from the culture. A bone flap removal procedure was performed, and the wound healed completely with primary closure. After another 1.5 years, a cranioplasty was performed to cover the bone defect using BoneSource® (Stryker, Kalamazoo, MI, USA), a calcium phosphate bone cement. Nonetheless, the scalp tissue over the BoneSource® was disrupted 2.5 years after cranioplasty. We removed the cement and debrided the overlying scalp tissues. The scalp defect was reconstructed using free LD muscle transfer and skin graft. No further wound complications have occurred for 12 years, and a secondary cranioplasty is planned in the near future.

## 4. Discussion

Late-onset radiation injuries can occur months or years after treatment. Although the mechanism is unclear, late-onset complications tend to occur in tissues with slow turnover rates [1].

RIF, a common finding of late-onset complications, has been well described in previous studies [2, 9]. Histopathologically, repetitive damage to the endothelial cells induces chronic inflammation, and active fibrosis begins in the extracellular matrix, which contains a high density of myofibroblasts.

ORN, another serious late-onset complication, is defined as radiation-induced delayed necrosis of the bone tissue that fails to heal over 3 months. The pathophysiology of ORN has not yet been clearly proven, but it does not usually occur at a radiation dose below 50–60 Gy, and its severity is known to be closely related to the total dose of radiation [10]. Our data showed that ORN occurred with a less intense radiation dose of 30 Gy, which may be due to the decreased tissue capability of bone flap recovery. Bone flaps created during craniotomy are vulnerable to radiation-induced damage as they are detached from the sources of blood supply, such as the dura, periosteum, and neighboring skull. Therefore, when ORN is suspected, complete removal of the bone flap along with debridement of the neighboring skull margin is important because the necrotic bone is highly susceptible to antibiotic-resistant microbial infection, which may lead to recurrent wound problems [11, 12]. Although accurate estimation of bone viability is not easy, imaging studies allow early diagnosis of ORN and better delineate the disease extent and are therefore recommended [13].

Wound closure should be attempted using the simplest possible method, according to the concept of a reconstructive ladder. If primary closure is not possible, a skin graft or a local flap should be performed. Skin grafting was not possible in most of our cases, as the wound did not provide a reliable bed for grafting. The local flap is the gold standard for treating moderate-sized scalp defects because it provides reliable hair-bearing soft tissue coverage. It is important to note that it has a low success rate in previously irradiated wounds, mainly because irradiated tissue has decreased perfusion and poor tissue elasticity due to RIF [10, 12]. We performed 5 free flap operations on 4 patients, where microanastomosis was done to the superficial temporal vessels. Many surgeons prefer the use of free flaps, and some even recommend them as the gold standard for treating irradiated scalp wounds [10, 12, 14, 15]. LD muscle and ALT fasciocutaneous flaps are frequently used for scalp reconstruction because they have sufficient flap volume with pedicles of considerable length and size suitable for microanastomosis. Surgeons should meticulously evaluate the condition of the recipient vessels when performing microvascular anastomosis in patients with a history of irradiation. If the vessels are in poor condition, recipient vessels should be identified in the previously irradiated area, or using an interposition vessel graft may be a reasonable alternative [16, 17].

Although previous reports have shown an increased postoperative complication risk when cranioplasty is performed in the field of preoperative irradiation, there was no significant difference according to the materials used for cranioplasties [8, 12]. Autologous bone grafts were not used in our cases as they are time-consuming with donor site morbidity and because the resorption rate is unpredictable, especially when grafted to previously irradiated fields [5]. We performed cranioplasties using BoneSource® in 3 patients at least 1 year after the scalp wound had stabilized. Nonetheless, two patients suffered from recurrent wound problems. In addition, cranioplasty material is a bio-burden, and mechanical tension and decreased perfusion from the bed can harm the overlying irradiated scalp tissue. Therefore, robust tissue coverage using free flaps is recommended when cranioplasty is scheduled.

We suggest a treatment protocol for the management of irradiated scalp wounds based on our single-center case series and a literature review (Figure 3). First, intracranial tumor recurrence should be ruled out. Tumors distort the surrounding tissue structure either physically or by releasing proteolytic enzymes. This may mimic radiation-induced tissue changes and, therefore, must be excluded [18]. If ORN is suspected, the bone flap and neighboring unhealthy tissues should be meticulously eradicated, followed by bone biopsy and antibiotic administration. If the scalp defect is small, primary closure or local flap placement can be performed. If the tissue defect exceeds 10 cm^2^ or if there is considerable wound tension, unhealthy scalp tissue should be widely excised, and coverage with a free flap should be performed. When a bone flap is removed with future plans to perform cranioplasty, it is highly recommended to debride the RIF scalp tissue and cover the defect with a robust free flap. LD muscle and ALT fasciocutaneous flaps are useful but can be changed according to the patient's clinical status or surgeon's preference. The recipient vessel can be selected as the most convenient site for anastomosis; however, preoperative vessel evaluation with Doppler or computed tomography angiography and intraoperative findings such as vessel size and pulsation should be considered.

## 5. Conclusions

Irradiation interrupts the normal wound healing process by inducing RIF in the soft tissue and ORN in the bone flap as a late complication. Reconstructive surgery for irradiated scalp wounds is associated with a high complication rate. Appropriate treatment of the bone flap and coverage with robust tissue are of utmost importance in scalp reconstruction.

## Figures and Tables

**Figure 1:** Removed titanium mesh, bone flap with ORN (ORN: osteoradionecrosis), and discarded scalp tissue showing characteristics of RIF (RIF: radiation-induced fibrosis).

**Figure 2:** Preoperative scalp wound and postoperative photo showing complete wound healing after LD muscle-free flap and STSG (LD: Latissimus dorsi; STSG: split-thickness skin graft). Published with the patient's consent.

**Figure 3:** Algorithms for surgical treatment of irradiated scalp wounds based on our clinical experiences and literature review.

**Table 1:** Patients' clinical information.

Pt. #	Sex	Age	Brain tumor	Loc	CTx	RTx (Gy/fx)	FB	Dur (years)	Operations	BFR	TNRS	Cx	CP	f/u (years)
1	F	27	GB	Rt T	O	54.0/30	LD	8	LF	X	1	MRSA	(-)	2
2	F	30	AA	Lt F	O	61.2/34	(-)	2.5	R+PC	O	1	(-)	(-)	1.5
3	M	70	AODG	Lt T	X	50.4/28	(-)	0.5	D+PC, LF+SG, R+FF	O	3	Pseudo	(-)	1.5
4	M	62	Mets	Lt F	O	30.0/10	SS	2	R+LF+SG	O	1	(-)	(-)	2.5
5	M	48	AM	V	X	61.2/34	(-)	14	LFx2, R (partial)+FF, R+FF	O	4	MRSE	(-)	1.5
6	F	24	GB	Lt FT	O	59.4/33	LD	1.5	(D+AD)x2, LF+SG	X	3	(-)	(-)	1.5
7	F	36	AA	Rt P	O	62.6/39	(-)	3.5	R+PC	O	1	MRSA	O	10
8	M	49	AODG	Lt F	O	59.4/33	(-)	11	D+PC, R+PC, LF, FF	O	4	Pseudo	(-)	2
9	M	38	GB	Rt F	O	61.2/34	LD	6	R+PC	O	1	MRSE	(-)	10
10	F	38	Olf NB	Lt F	O	54.0/30	(-)	2.5	D+PC, R+PC	O	2	MRSA	O	9
11	F	35	ODG	Rt F	O	59.4/33	(-)	1	R (partial)+PC D+LF, D+PC, FF, (D+PC)x2, R+PC	O	7	(-)	(-)	12
12	M	20	MG	Lt P	X	61.2/34	LD	1.5	R+PC	O	1	(-)	O	10.5
13	M	41	AODG	Rt FP	O	63.0/42	(-)	3.5	R+LF	O	1	SV	(-)	9

Pt.: patient; #: number; Loc: location; CTx: chemotherapy; RTx: radiotherapy; Gy: gray; fx: fraction; FB: foreign body; Dur: duration; BFR: bone flap removal; TNRS: total number of revision surgery; Cx: culture; CP: cranioplasty; f/u: follow-up; M: male; F: female; GB: glioblastoma; AA: anaplastic astrocytoma; AODG: anaplastic oligodendroglioma; Mets: metastasis; AMMG: atypical meningioma; Olf NB: olfactory neuroblastoma; ODG: oligodendroglioma; MG: meningioma; Rt: right; Lt: left; T: temporal; F: frontal; V: vertex; FT: frontotemporal; P: parietal; FP: frontoparietal; LD: Lyodura; SS: Surgisis; LF: local flap; R: removal of the bone flap; PC: primary closure; D: debridement; SG: skin graft; FF: free flap; AD: allodermis; MRSA: methicillin-resistant *Staphylococcus aureus*; Pseudo: *Pseudomonas aeruginosa*; MRSE: methicillin-resistant *Staphylococcus epidermidis*; SV: *Streptococcus viridans*.

## Data Availability

All the data supporting the results of this study (including those listed in the manuscript) is stored in the electronic medical records of Seoul National University Hospital.
